# The mechanism of hsa-miR-424-5 combining PD-1 through mTORC signaling pathway to stimulate immune effect and participate in Type 1 diabetes

This article has been retracted.

**DOI:** 10.1042/BSR20193800

**Published:** 2020-03-13

**Authors:** Guofeng Wang, Yongxin Yan, Zhichen Zheng, Tongyu Zhang

**Affiliations:** 1 Department of Endocrinology, The Affiliated Lianyungang Hospital of Xuzhou Medical University, The First People’s Hospital of Lianyungang, Lianyungang Clinical College of Nanjing Medical University, Lianyungang 222000, China; 2 Department of Gastrointestinal Surgery, The Affiliated Lianyungang Hospital of Xuzhou Medical University, The First People’s Hospital of Lianyungang, Lianyungang Clinical College of Nanjing Medical University, Lianyungang 222000, China

**Keywords:** hsa-miR-424-5p, immune effect, mechanism, mTORC signaling pathway, signal molecule, type 1 diabetes

## Abstract

In the present study, hsa-miR-424-5p mimic plasmid and hsa-mir-424-5p inhibitor plasmid were designed and injected into rats respectively, and miRNA control plasmid was also constructed. Models of Type 1 diabetes (T1D) were built. After successful modeling, the expression of hsa-miR-424-5p in lymphocytes was analyzed by RT-PCR. The expression of protein PD-1, T-bet, CXCR3, STING in Th1 lymphocytes and content of IGF-1 in islet tissue were analyzed by flow analysis. The protein levels of SHP2, Rheb, mTORC1, Rictor and Raptor in islet tissue were analyzed by Western blot. The results showed that hsa-miR-424-5p mimic group had the highest expression of hsa-miR-424-5p in lymphocytes. The expression of PD-1 was in hsa-miR-424-5p inhibitor > miRNA control > hsa-miR-424-5p mimic, while the expression of T-bet, CXCR3 and STING was in hsa-miR-424-5p mimic > miRNA control > hsa-miR-424-5p inhibitor. The expression of IGF-1 protein in hsa-miR-424-5p inhibitor group was the highest (32.08%) and hardly expressed in hsa-miR-424-5p mimic group (2.36%). The expression of SHP2, Rheb, mTORC1, Rictor and Raptor of insulin histoproteins were in hsa-miR-424-5p mimic group > miRNA control of > hsa-miR-424-5p inhibitor group, with statistical differences. It indicates that hsa-miR-424-5p binding PD-1 signaling molecules can stimulate the immune effect through the mTORC signaling pathway and participates in the pathogenesis of T1D.

## Introduction

Diabetes is the most common endocrine disease in almost all countries. It has a series of manifestations, such as chronic hyperglycemia. It was caused by the absolutely insufficient insulin secretion of islet β cells due to the destruction of their own immunity. Chronic hyperglycemia can lead to different organ damage and dysfunction, which lead to a series of complications. The most common complications of T1D include retinopathy, nephropathy, neuropathy and cardiovascular disease, which seriously affect the quality of life of patients [1,2]. With the change of lifestyle, the decrease in people’s physical activity and the increase in obesity, the number of diabetic patients is increasing year by year. Relevant research reports of International Diabetes Federation have estimated that the number of patients with diabetes will reach 642 million by 2040 [3]. Chronic diabetes has become an important issue of global public health concern. At present, the treatment of T1D is mainly insulin replacement therapy. However, long-term insulin replacement therapy often leads to blood glucose fluctuations, hypoglycemia, weight gain and other hazards [4,5].

Mammalian target of rapamycin (mTORC) is a kind of serine/threonine protein kinase that can regulate cell growth, metabolism, proliferation and survival by binding with other proteins to form two complexes: mTORC1 and mTORC2. mTORC1 and mTORC2 constitute signaling pathways with different upstream and downstream proteins to regulate cell growth, insulin, oxygen environment, energy, pressure, so as to activate translation, lipid synthesis, ribosomal biological transformation and inhibit autophagy [6,7]. Recent studies have shown that mTORC signaling pathway plays an important regulatory role in the occurrence and development of cerebrovascular diseases, autoimmune diseases and malignant tumors, but no study has been reported on the pathogenic mechanism of T1D. In addition, PD-1 belonged to the CD28/CTLA subgroup of transmembrane globulin and was expressed in activated TB lymphocytes [8,9]. It is a co-stimulatory molecule called T lymphocytes and is an immunosuppressive ligand. This project intends to research the related molecular mechanism of hsa-miR-424-5p combining with PD-1 signaling molecule to stimulate the immune effect through mTORC signaling pathway and participate in the pathogenesis of T1D.

## Experiment

### Materials

Streptozotocin (STZ) (Sigma); PBS (0.1 M, pH 7.0); 2.5% glutaraldehyde; Pancreatic enzyme; TRIzolRNA agent; DMEM/1640; FBS (Invitrogen); Trizol (Invitrgen); Cell culture dish: 6/12/48 plate (Thermo fisher); Sterile pipette: 5 ml/10 ml (Costar, U.S.A.); Liquid transfer gun: 10 μl/20 μl/200 μl/1000 μl (Eppendorf); centrifuge tube: 10 ml/50 ml (Thermo fisher); PCR instrument: Conventional PCR instrument, Western blotting instruments (Eppendorf); Confocal microscope (Olyplus, German); Flow meter BD; Ultra-thin slicer (LKB - V;JEOL Co.Japan); Transmission electron microscope (Jem-2000ex; JEOL Co.Japan).

### Methods

#### Construction of hsa-miR-424-5p mimic plasmid and hsa-miR-424-5p inhibitor plasmid

RNA was extracted from lymphocytes, and the target gene hsa-miR-424-5p was obtained by PCR. The upstream and downstream primers were added to EcoR I and BamH I’s enzyme digestion sites and incorporated into the carrier hsa-miR-424-5p mimic and hsa-miR-424-5p inhibitor plasmid, respectively. The gene sequencing identification of hsa-miR-424-5p mimic and hsa-miR-424-5p inhibitor was conducted by Shanghai Bioengineering Company. The results showed that the recombinant hsa-miR-424-5p mimic plasmid and hsa-miR-424-5p inhibitor plasmid had no gene mutation and met the experimental requirements.

#### Rat models of T1D

The research was operated in The First People’s Hospital of Lianyungang and Approval letter was obtained from The First People’s Hospital of Lianyungang. Thirty wistar male rats were purchased and fed with standard granular diet for one week. All rats were divided into three groups, 10 in each group. One group was injected with hsa-miR-424-5p mimic plasmid, the second group was injected with hsa-miR-424-5p inhibitor plasmid, and third group was injected with miRNA control plasmid. Then models of T1D were started. Fasting of rats at the day before the modeling, STZ, 0.1 mol/l, pH 4.2 citric acid buffer dissolved into 1% STZ solution, intraperitoneal injection according to STZ 60 mg/kg body weight, fasting blood glucose monitoring after injection. Blood glucose ≥ 16.65 mmol/l was considered as the molding standard. After successful modeling, the rats were anesthetized with 3% pentobarbital sodium (0.2 ml/100 g) and killed by cervical dissection. The abdominal aortic blood of the rats was immediately collected. At the same time, the islet tissue of the rats was collected and placed in the EP tube and stored in liquid nitrogen for further experiment [10].

#### Expression of hsa-miR-424-5p in lymphocytes

Expanded culture of rat lymphocytes was conducted, and RNA was extracted by cell lysis with TRIZol when cell density reached 95%. Total RNA was extracted according to Trizol method. About 0.05–0.1 g tissues were weighed first, and 1.0 ml of Trizol was added after EP tube and fully ground with Handy pestle. Total RNA was extracted from the homogenized tissue suspension in strict accordance with the Trizol instructions. The expression of hsa-miR-424-5p was measured RT-PCR.

#### Detection of Th1 lymphocyte content in blood

Rat lymphocytes cells were seeded on each well of 12-well plate at 37°C in an incubator containing 5% CO_2_ overnight. Next, the cells were incubated in medium containing DMEM without glucose for incubating 4 h, then the cells were washed with PBS for three times. The harvested cells were treated with trypsin/EDTA for 12 min, centrifuged at 1200 rpm for 3 min, and then the cell debris was suspended in 300 μl PBS. Fluorescence intensity of Th1 lymphocyte was measured using a FACS Aria I Spectral Analyzer (Becton Dickinson, U.S.A.).

#### Expression of PD-1, T-bet, CXCR3, STING in Th1 lymphocyte

Rat lymphocytes were centrifuged at 1100 rpm for 5 min, and the supernatant was removed. The cells were re-suspended, and a labeled antibody 20 μl that could bind integrin directly was added. The mixture was incubated at 37°C for 30 min, washed with 700 μl PBS, centrifuged at 1100 rpm, removed the supernatant, resuspended cells, added 1% paraformaldehyde PBS 500 μl, and detected by flow cytometry.

#### Immunohistochemistry analysis of IGF-1 expression in islet tissue

Immunohistochemistry staining was used to detect the expression of IGF-1 in islet tissue. Specific methods: the paraffin-embedded islet tissues of the rats were sectioned with a thickness of 4 μm. Immunohistochemistry two-step method was used for staining: the tissue sections were roasted at 65°C for 12 h, then dewaxed and hydrated. Endogenous peroxidase was inactivated by 3% hydrogen peroxide, and the specimens were washed with PBS for two times. Mouse anti-human IGF-1R was added and washed with PBS for two times. Then streptomycin working solution (labeled by horseradish peroxidase) was added and incubated at 37°C for 25 min. After completion, it was washed with PBS and stained with hematoxylin, then sealed with neutral chicle [11].

#### Western Blot analysis of SHP2, Rheb, mTORC1, Rictor and Raptor expression

Total proteins of tissue were extracted from tissue and 20 μg proteins were sampled. 5% concentrated gel and 12% isolated gel were prepared respectively to isolate proteins by SDS-PAGE. Objective and internal proteins were transferred to NC membrane, then closed with 5% skimmed milk powder sealing fluid for 2 h at room temperature. Rabbit anti Human primary antibody SHP2 (1:500), Rat anti Human primary antibody Rheb (1:500), Rat anti Human primary antibody, mTORC1, (1:500), Rat anti Human primary antibody Raptor (1:500) and Rat anti Human primary antibody β-actin (1:1000) were added and incubated at 4°C overnight. TBST washed four times, then HRP labeled Sheep anti Rat secondary antibody (1:5000) was added and incubated at 37°C for 1 h. TBST washed four times. Color was developed with ECL luminescent solution, protein bands were exposed by gel image analysis system, and images were photographed and quantitatively analyzed. The experiment was repeated three times.

### Statistical analysis

All experiments were repeated independently at least three times. One-way analysis of variance (ANOVA) was used to analyze the data, which was expressed as the mean ± standard deviation (S.D.). Statistical significance was defined as *P* <0.05.

## Results and discussion

### Rat models of T1D

During the experiment, the normal rats were in good condition, robust and normal autonomous activities. However, after 2 weeks, T1D symptoms such as listlessness, increased odor, polyphagia, polyuria and decreased body mass gradually appeared in the model mice. A total of 29 rats were successfully modeled with a success rate of 96.7%.

### Expression of hsa-miR-424-5p in lymphocytes

The expression of hsa-miR-424-5p of lymphocytes in the blood in hsa-miR-424-5p mimic group was higher than that of miRNA control (*P* <0.05), and much higher than that of hsa-miR-424-5p inhibitor group (*P* <0.01). The expression of hsa-miR-424-5p of lymphocytes was low in hsa-miR-424-5p inhibitor group compared with miRNA control (*P* <0.05) (Figure 1).

**Figure 1:** The expression of hsa-miR-424-5p in lymphocytes in different plasmid groups

### Detection of Th1 lymphocyte content in blood

Figure 2 showed that Th1 lymphocyte content in Q4 area was in hsa-miR-424-5p mimic > miRNA control > hsa-mir-424-5p inhibitor. Th1 lymphocyte mainly secrete cytokines such as IL-2, IFN-γ and TNF-β. Th1 lymphocyte mainly mediates cellular immune response and plays an important role in immune regulation in inducing organ-specific autoimmune diseases, organ transplant rejection and anti-infection immunity.

**Figure 2:** FCM analysis of Th1 lymphocyte content in blood

### Expression of PD-1, T-bet, CXCR3, STING in Th1 lymphocyte

Figure 3 showed that the expression of PD-1 was in hsa-miR-424-5p inhibitor > miRNA control > hsa-miR-424-5p mimic. However, the expression of T-bet, CXCR3, STING was in hsa-miR-424-5p mimic > miRNA control > hsa-miR-424-5p inhibitor.

**Figure 3:** Expression levels of PD-1, T-bet, CXCR3, STIN in Th1 lymphocytes in blood were analyzed by flow analysis

PD-1 is an important immunosuppressive molecule, which belongs to the immunoglobulin superfamily and is a membrane protein of 268 amino acid residues. It regulates the immune system and promotes self-tolerance by inhibiting the inflammatory activity of T cells. PD-1 expression was high in the hsa-miR-424-5p inhibitor group, which indicated that the immune system was suppressed. T-bet, CXCR3, STING were transcription factors of immune Th1 cells and Th2 cells, which participated in normal immune regulation and immune balance of T cells. It played an important role in the development of Th1 cells, so the expression levels of T-bet, CXCR3, STING were high in hsa-miR-424-5p mimic group. It indicated that mimic initiates immunity to participate in the regulation of diabetes.

### Immunohistochemistry analysis of IGF-1 expression in islet tissue

The staining results were determined as IGF-1 positive staining based on the tan or yellow granules of cytoplasm or cell membrane of epithelial cells in islet tissue. As could be clearly seen from the Figure 4, the miRNA control and hsa-miR-424-5p inhibitor group shows positive IGF-1. The expression of IGF-1 protein in miRNA control (14.72%) was higher than that of hsa-miR-424-5p mimic group (2.36%). A large number of IGF-1 mutations would lead to the deterioration of pancreatic islet cells. The expression of IGF-1 protein in miRNA control was highest in hsa-miR-424-5p inhibitor group (32.08%) compared the other two groups (*P* <0.01) (Table 1).

**Figure 4:** Immunohistochemistry analysis of positive expression of IGF-1 protein in islet tissue

**Table 1:** The expression of IGF-1 protein in islet tissue [*n*(%)]

	miRNA control	hsa-miR-424-5p mimic	hsa-miR-424-5p inhibitor
**Islet tissue (*n* = 3)**	14.72	2.36	32.08
**X^2^**	13.10	26.12	21.05
**P**	0.000	0.000	0.000

Insulin-like growth factor (IGF-1) is an important regulator of cell growth, which is widely present in human cytoplasm, extracellular and transmembrane regions, and is a glycoprotein transmembrane receptor. According to relevant research results, IGF-1 is abnormally expressed in breast cancer, ovarian cancer and other malignant tumor tissues and can promote the proliferation of tumor cells [12,13], but it has not been reported in the study on the mechanism of diabetes. In patients with diabetes, IGF-1 signal transduction can change the adhesion of cells and lead to malignant development of cells. Therefore, the diabetes complications will occur. Studies have shown that the mTORC pathway plays a key role in the metabolism of mitosis [14].

### Western Blot analysis of SHP2, Rheb, mTORC1, Rictor and Raptor expression

The expression of SHP2, Rheb, mTORC1, Rictor and Raptor in insulin tissue were shown in Figure 5. The expression of protein in hsa-miR-424-5p mimic group was higher than that of miRNA control (*P* <0.05), and much higher than that of hsa-miR-424-5p inhibitor group (*P* <0.01). Then, the expression of protein was low in hsa-miR-424-5p inhibitor group compared with miRNA control (*P* <0.05).

**Figure 5:** Protein level of SHP2, Rheb, mTORC1, Rictor and Raptor in different groups determined by Western blotting (mean ± SD, n=3) (**A**) Gray value; (**B**) Statistical analysis.

mTORC has long been considered as an suppressor of immune cells, but subsequent studies had shown that mTORC1 could promote the generation of Treg and enhance the immunosuppressive effect of T cells [15–17]. T1D is an autoimmune disease mediated by antigen presenting T cells. Previous studies had shown that inhibiting mTORC1 activity of CD4+T cells could inhibit Th1 and Th17 cell differentiation, promoted Th2 cell differentiation and improved immunity [18]. mTORC was composed of mTORC1 and mTORC2 [19]. mTORC1 was consist of mLST8, RAPTOR, DEPTOR and PRAS40. RAPTOR could combine with substrate of mTOR to make mTOR work [20]. mTORC2 was consisted of mLST8, RICTOR, DEPTOR, mSin1 and Protor1/2. RICTOR could maintain the stability of mTORC2 [21]. Zabo et al. [22] had shown that activation of mTORC1 signaling pathway could promote the immune response of T cells (Th1, Th17) and improved the immune response of the body. mTORC regulated the function of pancreatic β cells and inhibited GLP-1, a factor that promotes cell deterioration, thereby improving the complications of diabetes.

## Conclusion

Hsa-miR-424-5p can bind with PD-1 signaling molecules and stimulate immune effects through the mTORC signaling pathway to participate in the pathogenesis of T1D. However, there are some problems, such as small sample size, lack of clinical trials and so on, which still need to be further study.

## Abbreviations

IGF-1: insulin-like growth factor
mTORC: mammalian target of rapamycin
T1D: Type 1 diabetes
